# Application of Precise Positioning for Sputum Expectoration in ICU Patients with Pulmonary Infection

This article has been retracted.

**DOI:** 10.1155/2022/1395958

**Published:** 2022-01-29

**Authors:** Jing Wang, Mingyue Wang, Weiwei Li

**Affiliations:** Department of Critical Care Medicine, Shengjing Hospital of China Medical University, Shenyang City, 110004 Liaoning Province, China

## Abstract

**Objective:**

To determine the application value of precise positioning for sputum expectoration in intensive care unit (ICU) hospitalized patients with pulmonary infection (PI).

**Methods:**

A total of 183 patients with PI treated in the ICUs of Shengjing Hospital of China Medical University from June 2019 to June 2020 were divided into a control group (*n* = 91) and an observation group (*n* = 92), all of whom received conventional drug therapy. The control group was given routine nursing intervention, based on which, the observation group was supplemented with precise positioning for sputum expectoration. The 24-hour sputum volume, respiratory rate (RR), blood gas analysis indexes, inflammatory indicators, Clinical Pulmonary Infection Score (CPIS), Modified Medical Research Council (mMRC) dyspnea scale score, and quality of life (36-Item Short-Form Health Survey, SF-36) were observed in both arms before and after intervention. The incidence of adverse reactions was counted.

**Results:**

The observation group showed better mMRC scores than the control group (*P* < 0.05). Compared with the control group, the sputum volume, RR, and CPIS score were lower, and the SF-36 score was higher in the observation group 7 days after intervention (*P* < 0.05). After intervention, the oxygen saturation (SaO2) and partial pressure of oxygen (PaO2) were higher, while the carbon dioxide partial pressure (PaCO2), C-reactive protein (CRP), procalcitonin (PCT), and leukocyte count were lower in the observation group compared with the control group (*P* < 0.05). There was no significant difference in the incidence of complications between the two arms (*P* > 0.05).

**Conclusion:**

The application of precise positioning for sputum expectoration in nursing intervention of ICU patients with PI can alleviate the severity of PI and dyspnea, reduce inflammatory reaction, and improve the quality of life of patients.

## 1. Introduction

ICU patients generally have the characteristics of critical condition and rapid development, and they are more susceptible to pulmonary infection (PI) due to low immunity when receiving treatment, which may lead to the deterioration of their condition, resulting in poor treatment effect [1]. The etiology of ICU patients with PI is complicated, involving age, ICU stay time, mechanical ventilation treatment duration, tracheotomy or intubation, etc. [2]. As we know, ICU patients tend to keep secretions in the trachea and bronchi due to respiratory function decline and unresponsiveness, which makes PI difficult to cure for a long time. Therefore, the discharge of tracheal secretions is crucial for the treatment of PI [3]. This study mainly studies the excretion of tracheal secretions in ICU patients with PI, which is of great significance for improving the treatment effect and alleviating PI in such patients.

At present, atomization inhalation is often used for sputum aspiration. However, with this method, the sputum from deep bronchi can not be sucked out in time, and the ideal effect can be achieved only by repeated expectoration. While due to poor tolerance of ICU patients, repeated expectoration will inevitably increase the burden on the patient's lungs and affect the recovery of pulmonary function (PF) [4]. Research has pointed out that expectoration for PI can promote the recovery of PF [5]. Precise positioning for sputum expectoration is a nursing operation that dynamically combines the results of lung ultrasound examinations of patients to perform key sputum discharge nursing operations at the specific location and scope of sputum accumulation area, atelectasis area, or lung lesions, which can reduce the pulmonary burden and improve the respiratory function of patients. However, its application in ICU patients with PI is still in the exploratory stage. Accordingly, in this study, pulmonary ultrasound was used to accurately locate the sputum excretion site, and targeted chest physiotherapy was performed, aiming to explore the effect of this method on the inflammatory response and quality of life (QOL) of ICU patients with PI.

## 2. Materials and Methods

### 2.1. Clinical Data

The study population comprised 183 patients with PI treated in the ICUs of Shengjing Hospital of China Medical University from June 2019 to June 2020, including 91 cases in the control group and 92 cases in the observation group. There were 49 males and 43 females in the observation group, aged from 43 to 81 years, with a mean age of 60.80 ± 10.37 years. In the control group, the male to female ratio was 51 : 40, and the mean age was 59.01 ± 9.86 years (range: 41-78). There was no significant difference in the general data between the two arms (*P* > 0.05). This study was approved by the Ethics Committee of Shengjing Hospital of China Medical University.

### 2.2. Inclusion Criteria

Inclusion criteria are as follows: (1) ICU hospitalized patients with PI and length of stay > 2 weeks, (2) patients and their families voluntarily participated in this study and signed the informed consent, (3) CT examination of the lungs showed obvious infiltrative lesions, and (4) those with obvious moist rales in lung auscultation.

### 2.3. Exclusion Criteria

Exclusion criteria are as follows: (1) patients who cannot undergo ultrasound examination after thoracic surgery, (2) patients with severe thoracic deformity, (3) patients with massive subcutaneous emphysema, (4) patients with tuberculosis, lung tumors, or other lung diseases, and (5) patients who cannot cooperate with pulmonary rehabilitation treatment.

### 2.4. Methods

Patients in both groups were treated with conventional drugs, i.e., reasonably selected antibiotics for anti-infective treatment.

The control group was given routine nursing care: Sputum aspiration indications were determined by pulmonary auscultation of sputum sounds. After sputum aspiration, the patient was directly turned over for back percussion, followed by atomization inhalation. After completion, sputum aspiration was performed again.

The observation group was treated with precise positioning for sputum expectoration: Sputum aspiration indication was determined by pulmonary auscultation of sputum sounds. Pulmonary ultrasonography was performed after sputum aspiration and before the patient was turned over. According to the patients' PI and the ventilation of each area, the heavily infected parts were selected for percussion-on-back. The duration of back percussion was the same as that of the control group. Then, atomization inhalation was performed, after which sputum aspiration was given again. In both groups, airway clearance techniques such as postural drainage and tremor expectoration were combined to accelerate the drainage of airway secretions, maintain the patency of the respiratory tract, and improve the compliance of the thorax and lung.

### 2.5. Outcome Measures

(1) For primary outcome measures, the Clinical Pulmonary Infection Score (CPIS) [6], with a score ranging from 0 to 12, was used to evaluate the severity of PI of patients from 7 domains such as tracheal secretions, chest X-ray, and pulmonary infiltration. The higher the score, the more severe the PI. (2) For degree of dyspnea, seven days after intervention, the extent of dyspnea of patients was evaluated using the modified British Medical Research Council (mMRC) dyspnea scale [7]: Grade 0, generally no symptoms of dyspnea; Grade 1, symptoms of shortness of breath when hurrying on level ground or walking up a slight hill; Grade 2, walk slower than people of the same age because of breathlessness on level ground; Grade 3, stop for breath after walking a few minutes on level ground; and Grade 4, symptoms of breathless when dressing. (3) The 24-hour sputum volume and respiratory rate (RR) were compared between the two arms before and after intervention. (4) For QOL, the Short-form 36 Questionnaire (SF-36) [8] was used to evaluate the QOL of patients from 8 domains such as physical functioning, role-physical, and bodily pain. A higher score indicates a better QOL. (5) For blood gas analysis indexes, 3 mL of arterial blood was collected into heparin anticoagulation vacuum tubes to detect arterial oxygen saturation (SaO2), partial pressure of oxygen (PaO2), and partial pressure of carbon dioxide (PaCO2) using a blood gas analyzer (Shanghai Yuyan Scientific Instruments Co., Ltd., China, 57984). (6) For inflammatory factors, 5 mL of venous blood was collected from patients to measure the white blood cell count (WBC) and the levels of C-reactive protein (CRP) and procalcitonin (PCT). The WBC was detected using the Hitachi 7600 automatic biochemical analyzer, and the levels of CRP and PCT were determined by the enzyme-linked immunosorbent assay (ELISA) using human CRP ELISA kit and human PCT ELISA kit (Wuhan Fine Biotech Co., Ltd., EH0099, EH0341), respectively. The operation procedure was carried out in strict accordance with the instructions. (7) For complications, the incidence of atelectasis and other complications during hospitalization was statistically analyzed

### 2.6. Statistical Methods

Data were processed by the SPSS17 software (EasyBio (Beijing) Technology Co., Ltd., China). Enumeration data were represented by %, and *χ*^2^ test was used to compare the difference between groups. The measurement data were described as (±*s*) after normal test, and the difference between groups was analyzed by the *t*-test. The ranked data were compared by the *Z* test between groups. Paired *t*-test was used for comparison before and after intervention within the group. Statistical significance was defined as a *P* value < 0.05.

## 3. Results

### 3.1. Baseline Data

There were no significant differences in gender, age, average age, course of disease, educational level, drinking history, residence, and marital status between the two groups (*P* > 0.05) (Table 1).

### 3.2. Comparison of mMRC Scores between the Two Groups

The mMRC score was better in the observation group compared with the control group (*P* < 0.05) (Table 2).

### 3.3. Comparison of 24-Hour Sputum Volume, RR, and CPIS Scores between the Two Groups before and after Intervention

The sputum volume, RR, and CPIS score differed insignificantly between the two arms before intervention (*P* > 0.05). Seven days after intervention, the sputum volume decreased and was less in the observation group compared with the control group (*P* < 0.05); the RR and the CPIS score reduced in both arms and were lower in the observation group (*P* < 0.05) (Figure 1).

### 3.4. Comparison of SF-36 Scores between the Two Groups before and after Intervention

There was no significant difference in the SF-36 score between the two arms before intervention (*P* > 0.05). Seven days after intervention, the SF-36 score increased in both arms and was higher in the observation group (*P* < 0.05) (Table 3).

### 3.5. Comparison of Blood Gas Analysis Indexes between the Two Groups

Before intervention, the values of SaO2, PaO2, and PaCO2 had no significant difference between the two arms (*P* > 0.05). Seven days after intervention, SaO2 and PaO2 increased while PaCO2 decreased in both arms, with more significant alterations in the observation group compared with the control group (*P* < 0.05) (Table 4).

### 3.6. Comparison of Inflammatory Indicators between the Two Groups

The two arms had similar WBC and levels of CRP and PCT before intervention (*P* > 0.05). Seven days after intervention, the WBC and the levels of CRP and PCT reduced in both arms and were lower in the observation group compared with the control group (*P* < 0.05) (Table 5).

### 3.7. Comparison of Complication Rate between the Two Groups

Atelectasis occurred in 1 case in the observation group and 3 cases in the control group, with no significant difference between the two arms (*χ*^2^ = 0.262, *P* = 0.609).

## 4. Discussion

PI is a common respiratory disease, mostly manifested as symptoms such as dyspnea, cough, and expectoration. Due to the weakened PF of ICU patients, their ability of independent expectoration is reduced, resulting in the accumulation of sputum in the lungs, which may exacerbate PI [9]. Currently, the treatment of PI focuses on anti-infection and sputum removal [10]. More and more researchers have conducted research on sputum expectoration methods. For example, Kong et al. [5] reported that compared with simple lateral position ventilation, its combination with vibration sputum drainage can more significantly increase sputum excretion and improve the respiratory function of patients with acute respiratory distress syndrome (ARDS). In addition, Shi et al. [11] revealed that bronchoalveolar lavage combined with vibration sputum drainage had significantly better expectoration effect on patients with severe pneumonia and could also shorten the recovery time of patients. Precise positioning for sputum expectoration can be used to find the parts with severe PI through dynamic pulmonary ultrasound monitoring, which is helpful for clinical allocation of treatment time and nursing methods for atelectasis site according to the actual situation, as well as real-time evaluation of pulmonary rehabilitation treatment effect, thus alleviating dyspnea [12]. In this study, the observation group showed better mMRC scores than the control group. Moreover, SaO2 and PaO2 were higher, and PaCO2 was lower in the observation group compared with the control group. These results indicate that the application of precise positioning for sputum expectoration for ICU patients with PI can reduce the degree of dyspnea and hypoxia.

Precise positioning for sputum expectoration is a nursing operation that focuses on expectoration in the specific location and range of sputum accumulation area, atelectasis area, or lung lesions based on dynamic combination of lung ultrasound examination results, which can be targeted for sputum removal and more effectively remove sputum in the infected area, thus reducing the severity of PI. In addition, by reducing sputum accumulation, it can promote lung recruitment maneuvers and further improve PF [13, 14]. In this study, the sputum volume was less, and the respiratory frequency and CPIS score were lower in the observation group versus the control group after 7 days of intervention, indicating that the application of precise positioning for sputum expectoration for the nursing of ICU patients with PI could reduce the sputum excretion and the severity of PI.

Atomization inhalation, an extensively used sputum aspiration method, can promote the discharge of sputum from the lungs but cannot suck out the sputum with deep lesions. While as we know, sputum stasis is a risk factor leading to PI. Long-term sputum-stasis stagnation in the body will aggravate the severity of PI, prolong hospital stay, and reduce the QOL of patients [15, 16]. Na et al. [17] pointed out in their study that effective promotion of pulmonary sputum discharge can improve the function of pulmonary ventilation trachea and reduce clinical symptoms, thus improving the QOL of patients. The results of this study also revealed higher SF-36 scores in the observation group, which indicated that this intervention method could improve the QOL of patients. This is mainly because through precise positioning for sputum expectoration, the effect of sputum discharge can be enhanced, which can reduce the severity of dyspnea, promote the recovery of PF and improve the QOL.

CRP and PCT are diagnostic indicators of clinical infectious diseases. PCT can reflect the activity of systemic inflammatory reaction, while CRP is an acute inflammatory phase protein that is commonly used in the detection of inflammatory reaction [18]. It is reported that many patients with PI have increased secretion of pulmonary inflammatory factors, which will lead to substantial inflammation of alveolar cavity, interstitial lung, and airway. Sputum is an inflammatory secretion produced when the body has an inflammatory response, and sputum blocking the airway will lead to bronchial inflammatory edema, affecting the lung ventilation function [19]. Li et al. [20] pointed out that fiberoptic bronchoscopy for sputum aspiration in patients with PI can improve the efficiency of sputum excretion, thus reducing the inflammatory response. In this research, the observation group had lower WBC and levels of CRP and PCT, indicating that precise positioning for sputum expectoration in ICU patients with PI can reduce the inflammatory reaction, which is consistent with the abovementioned studies of Li et al. This is mainly related to the fact that precise positioning for sputum expectoration can promote the discharge of sputum from the infected site.

The novelty of this study is that we comprehensively evaluated and confirmed the feasibility and effectiveness of precise positioning for sputum expectoration in ICU patients with PI from various angles, such as the degree of dyspnea, 24-hour sputum volume before and after intervention, RR, severity of PI, QOL, blood gas analysis indexes, inflammatory indicators, and incidence of complications.

## 5. Conclusion

To sum up, the application of precise positioning for sputum expectoration in nursing intervention of ICU patients with PI can alleviate the severity of PI and dyspnea, reduce inflammation, and improve the QOL of patients.

## Figures and Tables

**Figure 1:** Comparison of 24 h sputum volume, respiratory rate, and CPIS score between the two groups before and after intervention. (a) The 24 h sputum volume of the observation group after 7 days of intervention was significantly lower than that before the intervention and the control group. (b) The breathing rate of the observation group after 7 days of intervention was significantly lower than that before the intervention and the control group. (c) The CPIS scores of the observation group after 7 days of intervention were significantly lower than those before the intervention and the control group. ^∗∗^*P* < 0.01.

**Table 1:** Baseline data of patients in the two groups (*n* (%), mean ± SD).

Variables	Control group (*n* = 91)	Observation group (*n* = 92)	*χ* ^2^/*t*	*P*
Gender			0.143	0.705
Male	51 (56.04)	49 (53.26)		
Female	40 (43.96)	43 (46.74)		
Age (years)			0.269	0.604
<60	48 (52.75)	45 (48.91)		
≥60	43 (47.25)	47 (51.09)		
Average age (years)	59.01 ± 9.86	60.80 ± 10.37	1.196	0.233
Course of disease (d)	7.45 ± 2.06	7.72 ± 2.39	0.818	0.414
Education level			1.266	0.747
Primary school	15 (16.48)	20 (21.74)		
Secondary school	35 (38.46)	33 (35.87)		
Junior college or undergraduate	26 (28.57)	22 (23.91)		
Bachelor degree or above	15 (16.49)	17 (18.48)		
History of drinking			2.016	0.156
No	55 (60.44)	46 (50.00)		
Yes	36 (39.56)	46 (50.00)		
Residence			2.292	0.130
Urban	60 (65.93)	70 (76.09)		
Rural	31 (34.07)	22 (23.91)		
Marital status			0.327	0.568
Single	22 (24.18)	19 (20.65)		
Married	69 (75.82)	73 (79.35)		

**Table 2:** Comparison of mMRC score between two groups (*n*).

Groups	*n*	Grade 0	Grade 1	Grade 2	Grade 3	Grade 4
Observation group	92	7	28	32	20	5
Control group	91	5	21	24	31	10
*Z*	5.081					
*P*	0.024					

**Table 3:** Comparison of SF-36 scores between two groups before and after intervention (point).

Groups	Time	Physical functioning	Role-physical	Bodily pain	General health	Vitality	Social functioning	Role-emotional	Mental health
Observation group (*n* = 92)	Before intervention	50.15 ± 3.50	52.52 ± 4.23	52.17 ± 5.15	50.86 ± 4.50	47.52 ± 5.09	52.17 ± 5.14	51.76 ± 5.38	49.27 ± 3.90
	7 days after intervention	62.27 ± 3.92^∗^	59.08 ± 4.39^∗^	59.62 ± 5.63^∗^	61.24 ± 5.07^∗^	57.42 ± 5.37^∗^	59.31 ± 5.29^∗^	59.24 ± 5.05^∗^	58.51 ± 4.35^∗^
	*t*	22.121	10.321	9.365	14.687	12.834	9.285	9.723	15.170
	*P*	<0.001	<0.001	<0.001	<0.001	<0.001	<0.001	<0.001	<0.001
Control group (*n* = 91)	Before intervention	51.07 ± 3.26	51.24 ± 4.17	51.92 ± 5.20	51.74 ± 4.35	49.05 ± 5.11	51.04 ± 5.32	50.09 ± 5.17	50.61 ± 4.18
	7 days after intervention	58.05 ± 3.85	56.21 ± 4.25	55.34 ± 5.57	58.09 ± 4.68	53.91 ± 5.29	55.68 ± 5.30	56.10 ± 5.09	55.83 ± 4.21
	*t*	13.199	7.963	4.281	9.481	6.303	5.894	7.902	8.393
	*P*	<0.001	<0.001	<0.001	<0.001	<0.001	<0.001	<0.001	<0.001

^∗^ *P* < 0.05 vs. the control group after intervention.

**Table 4:** Comparison of blood gas analysis indexes between two groups.

Groups	*n*	SaO2 (%)		PaO2 (mmHg)		PaCO2 (mmHg)	
		Before intervention	7 days after intervention	Before intervention	7 days after intervention	Before intervention	7 days after intervention
Observation group	92	90.18 ± 1.86	95.73 ± 2.14^#^	72.59 ± 3.16	87.13 ± 3.46^#^	51.57 ± 5.32	40.26 ± 3.82^#^
Control group	91	89.69 ± 1.80	94.17 ± 2.06^#^	73.20 ± 3.09	84.78 ± 3.51^#^	50.81 ± 5.24	43.19 ± 3.90^#^
*t*		1.811	5.023	1.320	4.561	0.974	5.134
*P*		0.072	<0.001	0.189	<0.001	0.332	<0.001

^#^ *P* < 0.05 vs. before intervention. SaO2: arterial oxygen saturation; PaO2: partial pressure of oxygen; PaCO2: partial pressure of carbon dioxide.

**Table 5:** Comparison of inflammatory indexes between two groups.

Groups	n	WBC (^∗^10^9^/L)		CRP (mg/L)		PCT (*μ*g/L)	
		Before intervention	7 days after intervention	Before intervention	7 days after intervention	Before intervention	7 days after intervention
Observation group	92	17.54 ± 2.38	10.31 ± 2.05^#^	8.16 ± 0.57	3.95 ± 0.41^#^	1.29 ± 0.20	0.51 ± 0.09^#^
Control group	91	16.92 ± 2.26	11.67 ± 2.08^#^	8.23 ± 0.63	4.16 ± 0.44^#^	1.24 ± 0.19	0.68 ± 0.11^#^
*t*		1.807	4.455	0.788	3.341	1.733	11.448
*P*		0.073	<0.001	0.432	0.001	0.085	<0.001

^#^ *P* < 0.05 vs. before intervention. WBC: white blood cell count; CRP: C-reactive protein; PCT: procalcitonin.

## Data Availability

The labeled dataset used to support the findings of this study are available from the corresponding author upon request.
